The article "Asymptomatic young male with ectopia cordis interna: A rare case report" was retracted in 2025. Reasons: plagiarized images; overlap with other authors' work; original data or images not available; unreliable results or conclusions.

# Asymptomatic young male with ectopia cordis interna: A rare case report

**DOI:** 10.1097/MD.0000000000043626

**Published:** 2025-07-25

**Authors:** Hashim Talib Hashim, Mohammedbaqer Ghuraibawi, Fatimah Abdullah Sulaiman, Batool S. Al-Aboudi, Zainab Ahmed Lateef, Ashraf Fhed Mohammed Basalilah, Bashar Hadi Shalan

**Affiliations:** a University of Warith Al-Anbiyaa, College of Medicine, Karbala, Iraq; b Al-Nassiryah Teaching Hospital, Nassiryah, Thi Qar, Iraq; c Faculty of Medicine, University of Kufa, Najaf, Iraq; d Hadhramaut Hospital, Hadhramaut, Yemen; e Anesthesia Techniques Department, College of Health and Medical Techniques, Al-Mustaqbal University, Babylon, Iraq.

**Keywords:** abdominal heart, congenital heart anomaly, ectopia cordis interna, incidental finding, rare condition

## Abstract

**Rationale:**

Ectopia cordis interna is a rare congenital condition that occurs when the heart is found within the abdominal cavity.

**Patient concerns:**

A 22-year-old Iraqi male with a chest infection presented to the clinic with a chest infection, during which the anomaly was incidentally discovered.

**Diagnoses:**

Although there are no clear symptoms, the anomaly can lead to potential risks during any abdominal procedures.

**Interventions:**

The patient got a chest X-ray for his infection, which revealed the anomaly.

**Outcomes and lessons:**

The case highlights the importance of early detection of this condition through imaging modalities and the need for focused research into its long-term implications and management strategies.

## 1. Introduction

Ectopia cordis Interna, also called Tin Man Syndrome, is a congenital condition that occurs when the heart is located within the abdominal cavity instead of the chest.^[1]^

A few cases of ectopia cordis interna have been reported in medical literature, and most of them are incidental discoveries during imaging studies or surgical procedures, which make it harder to detect it early. The cause of ectopia cordis interna is still unclear, but it is believed that it is caused by premature malformations in the thoracoabdominal wall and diaphragm. In the absence of other congenital anomalies or unrelated medical evaluations, the condition usually stays asymptomatic, such as in this case. Unintentional heart injuries during abdominal surgeries are a significant risk due to the placement of the heart inside the abdomen. Therefore, the report discusses how a 22-year-old boy with ectopia cordis interna was presented, diagnosed, and treated from the infection with an emphasis on the importance of recognizing this rare anomaly in clinical practice.^[2,3]^

## 2. Case presentation

A 22-year-old Iraqi male presented to the clinic with a persistent cough, mild shortness of breath, and fever lasting for 1 week. He stated that there was no chest pain, palpitations, or history of cardiovascular disease. There was no significant medical history, and his family history of congenital heart defects was negative. During the physical examination, the patient appeared to be well-nourished and not in any acute distress. With a temperature of 37.5°C, heart rate of 90 bpm, respiratory rate of 18 breaths per minute, and blood pressure of 120/80 mm Hg, the vital signs were in the normal range. No murmurs or evidence of cyanosis or clubbing were found in the heart during the cardiovascular examination. During the respiratory examination, there were scattered crackles on the right lower lung field, and the abdominal examination was unremarkable without any visible masses or tenderness. A mild infection was suggested by routine blood tests and the level of CRP When a chest X-ray was taken to evaluate the chest infection, it was found that there was an abnormal cardiac silhouette which is shown in Figure 1 raising suspicion of ectopia cordis interna. Contrast-enhanced computed tomography scans of the chest and abdomen were performed to confirm the presence of the heart within the abdominal cavity, confirming the presence of ectopia cordis interna as shown in Figure 2. There were no structural defects or signs of cardiac compromise in the heart. After administering a course of antibiotics, the patient successfully recovered from the chest infection and reported that it resolved without any complications. For his cardiac condition, no immediate intervention was necessary because he was asymptomatic. The patient stated that he is still asymptomatic without any signs or symptoms related to respiratory infections 3 months later. The staff advised him to seek immediate medical attention for any abdominal or surgical needs in the future, after receiving comprehensive counseling about his rare condition and risks.

**Figure 1.** Chest x-ray of the patient.

**Figure 2.** Abdominal CT scan. CT = computed tomography.

## 3. Discussion

Ectopia cordis interna is a rare congenital anomaly that occurs when the heart is placed inside the abdominal cavity instead of the chest1. It is also known as Tin Man Syndrome and derives its common name from the character in “The Wizard of Oz” who was famously without a heart.^[2]^ The classification of cases is usually based on the location of the heart relative to anatomical landmarks, such as the sternum, abdomen, thorax, or neck3, and there are only a few documented in medical literature.^[4]^

Notably, this anomaly was discovered in our patient during a chest infection evaluation, in consideration of the absence of any cardiovascular symptoms or diagnoses in the patient previously. This highlights the significance of imaging modalities, particularly ultrasound, as a main diagnostic tool, particularly for prenatal screening4. Ultrasound imaging can provide early detection of abnormalities, usually in the first or early second trimester, which allows for prompt identification in around 90% of reported cases. Diagnosis can now be made as early as 9 to 13 weeks’ gestation due to the integration of 2-dimensional and 3-dimensional sonography.^[5]^ The advantage of early recognition lies in managing potential physical and emotional complexities, especially in cases where elective termination may be considered.^[5]^ A combination of magnetic resonance imaging and fetal echocardiography is often used to monitor the progression of the condition and predict potential medical or surgical implications in cases of pregnancy.^[6]^

According to current literature, surgical interventions or postmortem examinations have been the most predictable methods of identifying ectopia cordis interna. According to previous reports, individuals with internal presentation often remain symptom-free until abdominal intervention becomes necessary, as indicated by the asymptomatic nature of this patient. The risk of inadvertent cardiac injury during abdominal surgeries is a major concern, so surgeons must be vigilant about this rare condition to prevent adverse outcomes during procedures like laparotomy.^[7]^

The development of ectopia cordis interna is believed to be caused by a failure to separate thoracic and abdominal cavities during early gestation. Although the exact etiology is still unclear, environmental factors and genetic mutations have been hypothesized as contributors. This malformation, which is usually sporadic, has been linked to chromosomal abnormalities such as trisomy 18, Turner syndrome, and 46, XX, 17q. The pathogenesis of this condition is influenced by embryonic migration and differentiation processes that start as early as the eighth day of embryonic life.^[8]^

Surgical intervention is widely accepted as the main treatment option for ectopia cordis interna, but a standardized surgical protocol has not yet been developed due to its rarity.^[7]^ The abdominal variant has a more favorable prognosis, but surgical efforts to correct thoracic and thoracoabdominal types have not been successful.^[8]^ However, there is agreement on the current recommendation for cautious monitoring and conservative management strategies, unless complications arise that require surgical intervention.

## 4. Conclusion

Ectopia cordis interna is a rare and captivating congenital condition, often discovered incidentally, as in this 22-year-old male who presented with a chest infection. Despite being asymptomatic, this condition underscores the necessity to proper preoperative planning. The importance of recognizing these anomalies in clinical practice is highlighted by this case and the need for further research to better understand the long-term implications and management of the condition.

## Acknowledgments

We thank all the authors for their contributions in the study.

## Author contributions

**Conceptualization:** Hashim Talib Hashim, Ashraf Fhed Mohammed Basalilah, Bashar Hadi Shalan.

**Data curation:** Hashim Talib Hashim, Batool S. Al-Aboudi, Ashraf Fhed Mohammed Basalilah.

**Formal analysis:** Hashim Talib Hashim, Fatimah Abdullah Sulaiman, Zainab Ahmed Lateef.

**Funding acquisition:** Hashim Talib Hashim, Bashar Hadi Shalan.

**Investigation:** Hashim Talib Hashim, Mohammedbaqer Ghuraibawi, Zainab Ahmed Lateef.

**Methodology:** Hashim Talib Hashim, Fatimah Abdullah Sulaiman.

**Project administration:** Hashim Talib Hashim, Fatimah Abdullah Sulaiman, Bashar Hadi Shalan.

**Resources:** Hashim Talib Hashim, Fatimah Abdullah Sulaiman.

**Software:** Hashim Talib Hashim, Batool S. Al-Aboudi.

**Supervision:** Hashim Talib Hashim, Bashar Hadi Shalan.

**Validation:** Hashim Talib Hashim, Mohammedbaqer Ghuraibawi, Ashraf Fhed Mohammed Basalilah.

**Visualization:** Hashim Talib Hashim, Mohammedbaqer Ghuraibawi.

**Writing – review & editing:** Hashim Talib Hashim, Mohammedbaqer Ghuraibawi, Bashar Hadi Shalan.

**Writing – original draft:** Mohammedbaqer Ghuraibawi, Fatimah Abdullah Sulaiman, Batool S. Al-Aboudi, Zainab Ahmed Lateef, Ashraf Fhed Mohammed Basalilah.
